RETRACTED

# Predictive Value of Serum Markers SFRP1 and CC16 in Acute Exacerbation of Chronic Obstructive Pulmonary Disease

**DOI:** 10.1155/2022/6488935

**Published:** 2022-08-02

**Authors:** Yewei He, Jian Yu, Dandan Zhu, Junlan Gao

**Affiliations:** Department of Critical Care Medicine, Second Hospital of Dalian Medical University, Dalian 116027, Liaoning, China

## Abstract

**Background:**

Chronic obstructive pulmonary disease (COPD) patients are particularly vulnerable to acute exacerbation, resulting in a huge socioeconomic burden.

**Objective:**

In this study, we evaluated the value of serum secreted frizzled-related protein 1 (SFRP1) and Clara cell-secreted protein (CC16) in predicting the risk of acute exacerbations in patients with COPD.

**Methods:**

The study included 123 COPD patients admitted to our hospital from May 2020 to June 2021, including 65 patients in stable stage (STCOPD group), 58 patients in acute exacerbation stage (AECOPD group), and 60 healthy volunteers (control group). Serum SFRP1 and CC16 levels were detected by enzyme-linked immunosorbent assay (ELISA). The receiver operating characteristics curve (ROC) analysis was performed to evaluate the sensitivity and specificity of serum SFRP1 and CC16 for predicting the risk of acute exacerbation in COPD patients.

**Results:**

The age among groups is significantly different, but there is no difference in the gender and body mass index (BMI). The level of serum SFRP1 in the AECOPD group was significantly higher than that in the STCOPD group and the control group, and the level of serum CC16 was lower than that in the STCOPD group and the control group. Serum SFRP1 was negatively correlated with forced expiratory volume in one second (FEV_1_)/forced vital capacity (FVC) (*r* = −0.473, *P* < 0.001). Serum CC16 was positively correlated with FEV_1_/FVC (*r* = 0.457, *P* < 0.001). The area under the curve (AUC), sensitivity, and specificity of SFRP1 for predicting the risk of exacerbation was 0.847 (95% CI: 0.775 to 0.920), 86.20%, and 80.00%. The AUC, sensitivity, and specificity of CC16 for predicting the risk of exacerbation were 0.795 (95% CI: 0.711 to 0.879), 74.10%, and 86.20%.

**Conclusions:**

These findings suggest that SFRP1 and CC16 may be useful serum markers for predicting the risk of exacerbation in COPD patients.

## 1. Introduction

Chronic obstructive pulmonary disease (COPD) is a general term for respiratory diseases that cause symptoms such as difficulty in breathing, cough, and sputum production [1]. COPD has a high incidence and a poor prognosis. According to WHO, COPD is currently the third leading cause of death in the world, causing 3.23 million deaths in 2019 [2]. Even COPD patients who adhere to a standardized inhaled pharmacologic therapy suffer from 0.5 to 3.5 episodes of acute exacerbations per year [3]. Airway inflammation and airflow limitation are aggravated in patients with AECOPD, which promotes different degrees of pulmonary function damage and even involves the circulatory system, resulting in respiratory failure and systemic inflammatory response. Frequent acute exacerbations reduce quality of life in COPD patients and increase the risk of mortality. The management strategy for COPD patients is the early detection and aggressive treatment of exacerbations. At present, the prediction approach of AECOPD relies entirely on the clinical manifestations and physicians' experience and is highly subjective. If there are objective indicators to evaluate the condition of COPD and predict the high risk of acute exacerbation, it can provide help for early clinical intervention in patients with high risk of acute exacerbation. In order to find biomarkers of AECOPD, the study samples were mainly derived from the respiratory tract and blood. During this study, we focused on blood-based biomarkers because blood samples are readily available.

RETRACTED

The pathogenesis of AECOPD remains unclear. Analyzing the molecular mechanisms involved in the pathogenesis of AECOPD will help monitor disease progression. Airway remodeling and airway inflammation are key components of airflow limitation throughout the progression of AECOPD [1]. Airway remodeling is a vicious cycle of airway wall damage and repair caused by chronic inflammation. The Wnt signaling pathway have been evidenced to be one of the key pathways involved in the development of chronic airway inflammation and airway remodeling. The Wnt pathway consists of Wnt proteins, frizzled (FZD) receptors, low-density lipoprotein receptor-related protein (LRP), and downstream molecules [4]. Wnt protein belongs to the family of secreted glycoproteins, which can activate the Wnt signaling pathway by specifically binding to the cell surface receptor FZD. Secreted frizzled-related protein 1 (SFRP1) is also a secreted glycoprotein. Differently, SFRP1 inhibits Wnt signaling through competitive binding with FZDs. Therefore, it is speculated that there is an important link between SFRP1 and COPD.

Clara cell-secreted protein (CC16) is mainly secreted by the Clara cells in the airway epithelium. CC16 is readily detected in the blood circulation and is specific for lung tissue. Serum CC16 levels are affected by the state of the Clara cells and the integrity of blood-gas barrier. CC16 exerts anti-inflammatory and antifibrotic biological activities. CC16 can inhibit the chemotaxis and phagocytosis of neutrophils and monocytes and can also inhibit the activity of phospholipase A2 (PLA2) to reduce the production of inflammatory mediators [5]. Low CC16 is not only a biomarker of airway pathology but may also be associated with the development of AECOPD and the progressive airway damage.

RETRACTED

SFRP1 and CC16 are associated with the development of COPD, but their roles in predicting AECOPD remain unclear. Our hypothesis is that SFRP1 and CC16 are important serum markers that predict high risk of AECOPD, allowing early exacerbations to be identified for early management. The aim of this study was to analyze whether they could serve as serum biomarkers for predicting COPD exacerbations.

## 2. Materials and Methods

### 2.1. Study Population

A total of 123 COPD patients with complete clinical data admitted to our hospital from May 2020 to June 2021 were selected as our research objects. This study included 65 patients with stable COPD (STCOPD, mean age was 63.13 years), 58 patients with acute exacerbation COPD (AECOPD, mean age was 67.53 years), and 60 healthy volunteers (control, mean age was 65.46 years). According to the diagnostic guidelines of the Global Initiative for Chronic Obstructive Lung Disease (GOLD), COPD is diagnosed when the FEV1/FVC is less than 70% along with typical symptoms and history of exposure to risk factors. Inclusion criteria for the STCOPD group included (1) patients with stable respiratory symptoms in the past 90 days; (2) no history of respiratory tract infection in the past 60 days; (3) no antibiotics, systemic hormones, or immunosuppressive therapy in the past 90 days. AECOPD patients were defined as those with aggravation of respiratory symptoms and the need for timely adjustment of treatment measures. Exclusion criteria for COPD patients as follows: (1) other lung diseases such as asthma, interstitial lung disease, lung cancer, and tuberculosis; (2) serious organic diseases; (3) mental illness or communication disorder. This study was carried out under the approval of the ethics committee of the Second Hospital of Dalian Medical University and conducted in accordance with the Helsinki Declaration. All participants have signed the informed consent.

### 2.2. Methods

Within 24 hours of admission, a morning blood sample was collected from each participant for serum. By retrieving the patient's electronic medical record, general clinical information of the patient, including name, age, and relevant medical history, can be obtained. The COPD patients were assessed using the COPD Assessment Test (CAT) and pulmonary function tests. Serum levels of SFRP1, CC16, interleukin-6 (IL-6), tumor necrosis factor-*α* (TNF-*α*), C-reactive protein (CRP), serum matrix metalloproteinase-9 (MMP-9), and vascular endothelial growth factor (VEGF) were detected by enzyme-linked immunosorbent assay (ELISA). ELISA kits for SFRP1 and CC16 were purchased from Abcam (Cambridge, UK). ELISA kits for IL-6, TNF-*α*, CRP, MMP-9, and VEGF were purchased from Biyuntian Biotechnology (Shanghai, China). All operations are carried out in strict accordance with the instructions.

RETRACTED

### 2.3. Statistical Analysis

SPSS 25.0 software (IBM SPSS 25.0, Armork, NY, USA) was used for statistical analysis, and measurement data were expressed as the means ± standard deviations (SD). If the data met a normal distribution, one-way ANOVA was used for comparison between groups. If the data presented a nonnormal distribution, a nonparametric test was used for between-group comparison. The enumeration data were expressed in the form of rate (%), and the chi-square test was used for comparison among the groups. Bivariate correlation analysis was performed using Pearson correlation analysis. The receiver operating characteristics curve (ROC) analysis was performed to evaluate the sensitivity and specificity of serum SFRP1 and CC16 for predicting the risk of acute exacerbation in COPD patients. A *P* value of <0.05 was considered to be statistically significant.

## 3. Results

A total of 123 COPD patients were included in this study, including 103 males and 20 females. Among the COPD patients, 65 cases were included in the STCOPD group, 58 cases were included in the AECOPD group, and 60 healthy volunteers were selected as the control group. The general clinical data of the study subjects are shown in Table 1. The age among the three groups is significantly different, but there is no difference in the gender and body mass index (BMI). Among COPD patients, 32 STCOPD and 35 AECOPD patients had a smoking history, and the smoking rate was higher than that of the control group. Patients in the AECOPD group had higher CAT scores and worse lung function, suggesting that the general condition of the patients was worse than the other two groups.

Table 2 is the comparison of serum marker levels in each group. We found that the level of SFRP1 in the AECOPD group was higher than that in the STCOPD group and the control group, while the level of CC16 was lower than that in the STCOPD group and the control group. We also examined common inflammatory markers and airway remodeling-related markers. IL-6, TNF-*α*, CRP, MMP-9, and VEGF in the AECOPD group were significantly higher than those in the STCOPD group and the control group.

Then, the relationship between the level of SFRP1 and CC16 and FEV_1_ and FEV_1_/FVC in COPD patients were performed by Pearson's correlation analysis. As demonstrated in Figures 1(a) and1(b) and Figures 2(a) and 2(b), serum SFRP1 was negatively correlated with FEV_1_ and FEV_1_/FVC (*r* = −0.563, −0.473, *P* < 0.001). Serum CC16 was positively correlated with FEV_1_ and FEV_1_/FVC (*r* = 0.500, 0.457, *P* < 0.001).

RETRACTED

To further explore the value of serum SFRP1 and CC16 levels in predicting the risk of exacerbations in COPD patients, we established an ROC analysis (Figure 3). As shown in Figure 2 and Table 3, the critical value of SFRP1 was 115.99 pg/mL, the sensitivity was 86.20%, the specificity was 80.00%, and the Youden index was 0.662. The critical value of CC16 was 62.11 pg/mL, the sensitivity was 74.10%, the specificity was 86.20%, and the Youden index was 0.603. The AUC of SFRP1 combined with CC16 (0.911) is higher than that of the SFRP1 (0.847), which is higher than the AUC of the CC16 (0.795).

## 4. Discussion

The prevalence of COPD is still increasing year by year, and acute exacerbation is a serious clinical adverse event in COPD patients. In COPD patients with repeated acute attacks, the lung function deteriorates rapidly, the quality of life decreases, the hospitalization rate increases, and the mortality rate increases significantly, which seriously threatens the life and health of COPD patients [6, 7]. To reduce the number of exacerbations in STCOPD patients, a variety of drugs have been developed. However, there are still a large number of patients with standardized treatment who experience 2 or more acute exacerbations per year. At present, prediction of acute exacerbation risk mainly relies on doctors' judgment on patients' clinical symptoms [8], which is highly subjective. If there are objective biomarkers that can predict patients at high risk of acute exacerbation, it will be of great significance for monitoring disease progression and early intervention for the outcome of high-risk patients.

The pathogenesis of COPD has not been fully elucidated. The mainstream view holds that airway inflammation and airway remodeling are the key links in causing airflow limitation, which run through the progression of COPD. The abnormal increase of specific inflammatory cells and cellular mediators in different parts of lung tissue can cause structural changes after repeated injury and repair of airways and lung parenchyma. Controlling and reducing the degree of lung function reduction in patients with AECOPD can help improve the prognosis and quality of life of patients.

Many signaling pathways are involved in the pathogenesis of COPD, and Wnt signaling is one of the major signaling pathways [9]. In emphysema patients, Wnt signaling activity has been reported to be suppressed, and target gene expression is reduced [10]. And, this change leads to the weakening of emphysema. SFRP1 is an important member of the secreted frizzled-related protein family. SFRP1 is mainly distributed in lung tissue and is closely related to airway development and airway morphological changes. SFRP1 is the largest family of the Wnt signaling pathway antagonists and can inhibit the Wnt pathway by competitively binding to FZD on the cell membrane [11]. Previous studies have shown that SFRP1 is highly expressed in the lung tissue of patients with emphysema [12]. But what we do not know is the changes of serum SFRP1 levels in COPD patients. The results showed that the serum SFRP1 level in COPD patients was higher than that in healthy volunteers, and the SFRP1 level in AECOPD patients was higher than that in STCOPD patients. The results suggest that SFRP1 may be involved in the occurrence and progression of COPD.

RETRACTED

Clara cells are peripheral airway progenitor cells that are susceptible to damage and diminished by chronic inhalation irritants [13]. Patients with COPD have reduced Clara cells [14]. CC16 is a lung tissue-specific protein secreted by airway Clara cells, and serum CC16 can be detected by concentration difference from the epithelial lining fluid of lung cells into serum [15]. Serum CC16 levels have been confirmed in assessing lung epithelial cell permeability and Clara cell integrity. CC16 has strong anti-inflammatory and antifibrotic biological activities. In the early stage of acute lung injury, serum CC16 concentration is elevated due to damage to the lung-blood barrier [16]. In chronic lung injury, the decrease in the number of Clara cells results in decreased secretion of CC16 due to damage to the airway epithelial cells [17]. Airway remodeling, decreased Clara cell numbers, etc., are the theoretical basis for the association of CC16 with COPD. The research results of Rong et al. [18] showed that compared with healthy controls, serum CC16 levels were downregulated in STCOPD patients.

Our results found that serum CC16 levels in AECOPD patients were significantly lower than those in STCOPD patients and healthy controls. The level of CC16 was positively correlated with lung function and negatively correlated with the severity of the patient's disease. The research of Rizwan et al. [19] supports the findings of this study. The mechanism may be due to the destruction of Clara cells by acute aggravated airway inflammation, resulting in a decrease in secreted proteins and a decrease in the concentration of CC16 in peripheral blood. The CC16 concentration of patients in the stable phase increased to a certain extent. Changes in serum CC16 concentrations occurred earlier than changes in clinical lung function [20], suggesting that serum CC16 may be a serum marker for predicting the risk of acute exacerbations in COPD patients.

RETRACTED

In this study, the levels of inflammatory markers IL-6, TNF-*α*, and CRP [21, 22] and airway remodeling-related markers MMP-9 and VEGF [23] were detected. Elevated levels of inflammatory factors indicate that there are inflammatory responses and immune response imbalances in COPD patients [24]. The results of this study showed that IL-6, TNF-*α*, CRP, MMP-9, and VEGF in the AECOPD group were significantly higher than those in the STCOPD group and the control group. Further analysis found that SFRP1 was associated with MMP-9 and VEGF. This suggests that SFRP1 may promote airway remodeling in COPD patients.

Combination of SFRP and CC16 found that AUC was greater than these single markers in predicting exacerbation risk. The results show that the combined detection of SFRP1 and CC16 has more predictive value than a single indicator. In conclusion, serum SFRP1 levels were significantly increased, while CC16 levels were significantly decreased in AECOPD patients compared to STCOPD patients. SFRP1 and CC16 may be useful serum markers for predicting the risk of exacerbation in COPD patients.

## Figures and Tables

**Figure 1:** Correlation of SFRP1 with FEV1 and FEV1/FVC. (a) Correlation analysis between the level of SFRP1 and FEV1 in COPD patients. (b) Correlation analysis between the level of SFRP1 and FEV1/FVC in COPD patients.

**Figure 2:** Correlation of CC16 with FEV1 and FEV1/FVC. (a) Correlation analysis between the level of CC16 and FEV1 in COPD patients. (b) Correlation analysis between the level of CC16 and FEV1/FVC in COPD patients.

**Figure 3:** Receiver operating curves of SFRP1 and CC16 predicting the risk of AECOPD.

**Table 1:** General clinical data of the study objects.

Items	Control (*n* = 60)	STCOPD (*n* = 65)	AECOPD (*n* = 58)	*P* value
Age, years, mean (SD)	65.46 ± 8.53	63.13 ± 9.28	67.53 ± 8.29	0.023
Gender, male, (*n*, %)	49 (81.67)	52 (80.00)	51 (87.93)	0.474
BMI, kg/m^2^, mean (SD)	23.01 ± 2.27	22.81 ± 1.98	22.64 ± 2.11	0.638
History of smoking (*n*, %)				0.002
Yes	21 (35.00)	32 (49.23)	35 (60.34)	
No	39 (65.00)	33 (50.77)	23 (39.66)	
COPD duration, years, mean (SD)	NA	8.81 ± 2.41	10.23 ± 3.27	0.007
Lung function indexes, mean (SD)				
FEV_1_ (% predicted)	98.54 ± 5.03	70.14 ± 11.38	62.33 ± 13.26	<0.001
FEV_1_/FVC (%)	83.29 ± 3.06	64.17 ± 5.34	57.87 ± 6.14	<0.001
CAT score, mean (SD)	NA	20.15 ± 3.58	27.78 ± 4.23	<0.001
Arterial blood gases, mean (SD)				
PaO_2_ (mmHg)	83.69 ± 4.44	57.23 ± 6.36	56.11 ± 7.03	<0.001
PaCO_2_ (mmHg)	38.26 ± 5.31	43.09 ± 7.48	44.63 ± 6.52	<0.001

STCOPD, stable chronic obstructive pulmonary disease; AECOPD, acute exacerbation of chronic obstructive pulmonary disease; BMI, body mass index; FEV1, forced expiratory volume in the first second; FVC, forced vital capacity; CAT, the COPD assessment test.

RETRACTED

**Table 2:** Comparison of serum indexes in each group.

Parameters, mean (SD)	Control	STCOPD	AECOPD
SFRP1, pg/mL	58.85 ± 4.91	112.02 ± 19.46^a^	142.15 ± 20.13^a,b^
CC16, pg/mL	99.53 ± 6.80	70.09 ± 10.79^a^	54.43 ± 13.59^a,b^

Inflammatory markers			
IL-6, pg/mL	83.11 ± 13.62	123.84 ± 13.26^a^	140.96 ± 9.37^a,b^
TNF-*α*, ng/L	8.10 ± 2.30	15.67 ± 2.60^a^	26.34 ± 3.56^a,b^
CRP, mg/L	2.40 ± 0.53	6.22 ± 1.37^a^	12.00 ± 2.20^a,b^

Others			
MMP-9, *μ*g/L	74.29 ± 6.44	118.77 ± 7.20^a^	149.75 ± 9.44^a,b^
VEGF, mg/L	21.13 ± 3.39	35.59 ± 4.13^a^	62.42 ± 11.93^a,b^

*Note. *a*P* < 0.001 versus control group; b*P* < 0.001 versus STCOPD group.

**Table 3:** Sensitivity, specificity, and cutoff point of SFRP1 and CC16.

Parameter	AUC (95% Cl)	Cutoff	Sensibility	Specificity	Youden index
SFRP1	0.847 (0.775–0.920)	115.99	0.862	0.800	0.662
CC16	0.795 (0.711–0.879)	62.11	0.741	0.862	0.603
SFRP1 + CC16	0.911 (0.864–0.958)	125.69	0.966	0.677	0.642

## Data Availability

The data used to support the findings of this study are available from the corresponding author upon request.
